RETRACTED

# Mathematical Modelling and Prediction of the Effect of Chemotherapy on Cancer Cells

**DOI:** 10.1038/srep13583

**Published:** 2015-08-28

**Authors:** Hamidreza Namazi, Vladimir V. Kulish, Albert Wong

**Affiliations:** 1 School of Mechanical and Aerospace Engineering, Nanyang Technological University, Singapore; 2 School of Mechanical and Aerospace Engineering, Nanyang Technological University, Singapore; 3 Department of Radiotherapy, Oncology and Palliative care, Sarawak General Hospital, Kuching, Malaysia

## Abstract

Cancer is a class of diseases characterized by out-of-control cells’ growth which affect DNAs and make them damaged. Many treatment options for cancer exist, with the primary ones including surgery, chemotherapy, radiation therapy, hormonal therapy, targeted therapy and palliative care. Which treatments are used depends on the type, location, and grade of the cancer as well as the person’s health and wishes. Chemotherapy is the use of medication (chemicals) to treat disease. More specifically, chemotherapy typically refers to the destruction of cancer cells. Considering the diffusion of drugs in cancer cells and fractality of DNA walks, in this research we worked on modelling and prediction of the effect of chemotherapy on cancer cells using Fractional Diffusion Equation (FDE). The employed methodology is useful not only for analysis of the effect of special drug and cancer considered in this research but can be expanded in case of different drugs and cancers.

Cells production and die are regulated in human body in an orderly way. But in case of cancer, the division and growth of cells is out of control. In this manner, the damaged cells start to occupy more and more space in a part of body and so they expel the useful healthy cells. By this way that part of body is called tumor. So fighting with these cancer cells and changing the way of their production and accumulation is a critical issue in medical science.

Scientists have developed different methods for treatment of cancer. Some of these methods are surgery, chemotherapy, radiation therapy, hormonal therapy, targeted therapy and palliative care. Employing the less-invasive methods have always had critical role in patient treatment. Chemotherapy as a method for cancer treatment deals with application of drugs affecting the cancer cell’s ability to divide and reproduce. The drug makes the cancer cells weak and destroys them by directly applying to cancer site or through the bloodstream.

During years some researchers have worked on mathematical modelling of the effect of chemotherapy on cancer treatment. Some researchers employed different types of differential equations for modelling of the effect of chemotherapy on cancer treatment. For instance, Pillis *et al.* developed a mathematical model based on a system of ordinary differential equations which analyses the cancer growth on a cell population level after using chemotherapy^1^. Despite the overall success of this mathematical model, it couldn’t explain the effects of IL-2 on a growing tumour. So, in another work Pillis *et al.* updated their model by introducing new parameters governing their values from empirical data which are specific in case of different patients. The new model allows production of endogenous IL-2, IL-2-stimulated NK cell proliferation and IL-2-dependent CD8^+^ T-cell self-regulations^2^. In another work, using a system of delayed differential equations, Liu and Freedman proposed a mathematical model of vascular tumor treatment using chemotherapy. This model represents the number of blood vessels within the tumor and changes in mass of healthy cells and competing parenchyma cells. Using the proposed model they considered a continuous treatment for tumor growth^3^. See also^4^,^5^. In a closer approach some researchers specially focused on mathematical modelling of the diffusion of anti-cancer drugs to cancer tumor^6^,^7^,^8^,^9^,^10^,^11^.

RETRACTED

Beside all the works done on mathematical modelling of cancer treatment using chemotherapy, no work has been reported which analyse and model this treatment by linking between DNA walk and drug diffusion. In this research we model the response of tumor to anti-cancer drug. For this purpose we consider the diffusion of the drug in solid tumor. This diffusion will cause the damaged cells die and thus healthy cells appear.

In the following first we talk about DNA walk as a random multi fractal walk. After that we discuss about chemotherapy and diffusion of drug in tumor. By considering these two topics we start to develop the Fractional Diffusion Equation (FDE) which maps the effect of drug diffusion on DNA walk. The result and discussion remarks are brought in last sections.

## Method

### Chemotherapy and Diffusion

Chemotherapy as a famous method of cancer treatment is the application of drug to patients. Different types of drugs can be used in chemotherapy based on the type of cancer. A single drug or combination of drugs can be used simultaneously in chemotherapy. In fact drugs use a programmed form of cell death known as apoptosis in order to kill cancer cells. Cancer cells may respond to chemotherapy agents with different rates. Different types of drugs employ different methodologies to fight cancer cells. In this research we consider the application of anti-cancer drugs to the cancer tumor through blood stream. Coming closer to the tumor, drug diffuses to the tumor through the capillary which is surrounded by tumor. In fact, distribution of cancer drugs in tumor tissue depends on drug delivery, drug diffusion and drug consumption as it is shown in Fig. 1^12^.

RETRACTED

According to Fig. 1, the drug diffuses to the tumor through capillary. Then, the drug is consumed by tumor which affects the cancer cells’ behaviour in production and die. It is noteworthy to mention that different drugs travel in blood vessel with different velocities and accordingly diffuse in tumors with different diffusion rates. In a similar manner the consumption of drugs are different in case of different types of tumors.

In this research we focus on anti-cancer drugs that travel through blood stream to reach the tumor and diffuse in it.

### DNA Walk Analyses

It is known that DNA of the cell’s chromosome consist of four letters which are A, C, G and T that are bases adenine, cytosine, guanine and thymine respectively. The DNA sequence can be written in the form of numbers by converting A, C, G, T to 2, 3, 4, 1 respectively. By employing a popular mathematical method we can generate the DNA walk of genome. In this method first the DNA text is converted to a binary sequence and then DNA walk is generated by cumulative variables^13^.

It is known that DNA walk is a random walk and accordingly fractal. So, the concept of fractal dimension can be defined for this motion in order to talk about its complexity. In the research done by Namazi and Kiminezhadmalaie, it was shown that DNA walk is not defined by only a single fractal dimension but it has a spectrum of fractal dimensions^13^.

They proved that the analysis of fractal dimension and Hurst exponent spectra is a key tool for analysis of DNA walk complexity and predictability respectively. In fact, DNA walk in case of cancer cells is different from the DNA walk is case of normal cells. As they wrote, the DNA walk is case of cancer cells shows higher degree of fractality (bigger values of the fractal dimension) and less degree of predictability (smaller values of the Hurst exponent) compared to the DNA walk for normal cells.

In the next section by considering the DNA walk as a multi fractal series we make a relationship between the diffusion of anti-cancer drugs and DNA walk using Fractional Diffusion Equations (FDE).

### Fractional Diffusion Model of DNA Walk

Here in order to develop our model first we talk about the diffusion phenomena. As it was mentioned before, here we consider the diffusion of anti-cancer drug in tumor. The drug is delivered to patient’s body through intravenous infusion directly into the blood stream. After that the drug travels to the tumor and diffuses from the capillaries into tumor tissue as it shown in Fig. 1. So we can start from the well-known diffusion equation:



Equation (1) is the diffusion equation where *D* is the diffusion coefficient for diffusion of the property *F* (drug) in the medium (tumor). This diffusion process can be studied for fractals. Considering DNA walk as a fractal series, then the Fractional diffusion equation^14^ can be developed:



In this equation , *C* is the speed of propagation, *l* is nucleotide distance and *H* is the Hurst exponent. Hurst exponent as indicator of process memory falls in range 0 ≤ *H* ≤ 1 and bring the predictability into account. If 0 < *H* < 0.5, the process is anti-persistent and when 0.5 < *H* < 1 the process is persistent. Please note when *H* = 0.5 the process is completely random.

RETRACTED

In this research we want to show that DNA walks as multi fractal series which represent a transient record in the form of a random walk process, can be modelled by the solution of the Fractional Diffusion Equation (Equation 2), where *F* stand for purine-pyrimidine displacement in DNA walk plot. We aim to show the effect of diffusion of anti-cancer drug to tumor and killing the damaged cells can be modelled by this equation. If so, we made a relationship between diffusion on one side and fractal DNA walk on the other side using Equation (2).

In this research *C* is speed of drug delivery to tumor which is a finite quantity and equals to blood velocity. The term *D*, the diffusion coefficient, as the property of tumor, is related to tumor’s resistance to the anti-cancer drug as it deliver over the tumor. Equation (2) is valid for *l* ≥ 0 with the initial condition *F*(*x*, 0) = *F*_0_ at *l* = 0, and the boundary condition:



in the case of infinite domain. It is noteworthy *η* is the spatial variable. Here we used the Oldham and Spanier method^15^ in order to solve Equation (2).

By introducing the excess value , we have the following initial condition on 



By applying the Laplace transform to Equation (2) with respect to *l*:



In this equation *s* is the Laplace transform variable, and *Y* is the Laplace transform of .

The general solution of Equation (5) is:



In this equation *B*_1_(*s*) and *B*_2_(*s*) are two arbitrary functions. As the solution is to be bounded for all *η*, *B*_2_(*s*), must be identically zero, so:



Then we differentiate this equation respect to *η*:



By comparing (7) and (8), we eliminate *B*_1_(*s*), then:



By taking the inverse Laplace transform of this equation:



Equation (10) is in terms of fractional derivative of order −*H* with respect to *l*.

Considering the fractional derivative^14^:



In this equation, Γ(*α*) is the Gamma function. In order to bring the presence of drug in our formulation we model it as flux, *φ*, through Fick’s Law:

Then:



This equation makes a relationship between *F*(*η*, *l*), as the DNA walk fluctuation, and anti-cancer drug as the external influence acting on the tumor, . This equation is valid for every location within the tumor (including the boundary).

RETRACTED

It follows from equation (13) that the value of *F*, on the average, increases with *l* according to the power law as *l*^*H*^, considering the fluctuations are small in comparison with the averaged influence.

In this research  is modelled by a Gaussian pulse:



In Equation (14) l* is the moment, at which the Gaussian pulse has its maximum which is . *σ* stands for standard deviation of the Gaussian pulse. Please note that base on the strength of anti-cancer drug and its dose, the parameters in Equation (14) can have different values.

Figure 2 shows the real damaged DNA walk and solution of Equation (13) (after *l* = 4.2) for arbitrary values of parameters. As it can be seen in this figure the application of anti-cancer drug in this plot is clear by a sudden upward deflection. After this deflection the value of purine-pyrimidine displacement changes according to power law as the result of Equation (13).

Figure 3 shows the Hurst exponent plot for the DNA walk (pre- and post-application of drug) shown in Fig. 2. As it can be seen the application of anti-cancer drug in this plot is shown by a sudden upward deflection which increases the values of the Hurst exponent. After this deflection the values of the Hurst exponent continue to decrease again.

Figure 4 shows the Fractal spectrum plot for the DNA walk (pre- and post-application of drug) shown in Fig. 2. As it can be seen the application of anti-cancer drug in this plot is shown by a sudden downward deflection which decreases the values of the Fractal dimension and decreases the complexity of DNA walk. After this deflection the values of the Fractal dimension continue to increase again.

### Analysis

As it is known the human DNA is same in the body. As it was mentioned before, in case of cancer, the DNA walk is changed to be more fractal and less predictable for cancer cells compared to normal healthy cells. When human gets a special type of cancer, like lung cancer, only that organism’s cells converted to cancer cells and make a tumor by combining together and not die. So, other parts of the body still have normal cells. Thus, in this case two types of DNAs can be found in human body. We use this phenomenon as a key tool for our analysis. In fact, we take the DNA walk of cancer cells as input to Fractional Diffusion Equation (FDE). Then, after applying the anti-cancer drug to the cancer cells, they will die, and by replacing with normal cells the DNA will be changed to normal DNA. This normal DNA is like the DNA of other healthy cells in human body. So we know what should be the outcome of drug application. The model output should be similar with the normal DNA walk. In order to test the strength of model we compute the Hurst exponent and Fractal dimension spectra for the governed DNA walk from the model. These spectra should be similar with the Hurst exponent and Fractal dimension spectra for the DNA walk taken from healthy cells of other parts of body.

RETRACTED

### Data Collection

In this research the experiments have been done on 50 patients (25 men and 25 women with age in the range of 30 ± 2 years old) with histologically confirmed small cell lung cancer that all of them were smoker with the same height and weight. It is noteworthy that all patients were in early step of lung cancer. Patients didn’t receive chemotherapy or radiotherapy before their recruitment.

At first, each subject was interviewed by a physician to describe the nature of experiments for them. Informed consent was obtained from all subjects after the nature of the study was fully explained. All procedures (experiments, etc.) were approved by the Internal Review Board of the University and the approval for experimentation involving subjects was issued by Sarawak General Hospital and the university. The methods used in this research were carried out in “accordance” with the approved guidelines. It is noteworthy that the identity of all subjects remains confidential.

In the first step of experiment, the DNA samples were collected from the hairs of patients. For this purpose 10 hairs were plucked from the back of the patient’s shoulder. The DNA extraction was done using the method described in^16^. It is noteworthy that DNA which was collected in this step belongs to normal cells.

In the second step of experiment, the cancer DNAs was collected from patients with lung cancer. In fact, tumors shed nucleic acids (DNA or RNA) into the blood stream. So, the plasma can be used as the source of tumor DNA^17^. Scientists believe that plasma DNA is of tumor origin as its genetic alterations are similar with the corresponding primary tumors^18^. So in this research in order to take the DNA non-invasively we use the plasma as the source of lung cancer DNA. For this purpose we employed the similar methodology used by Weber *et al.*^19^. In this research we used 2 mL of the plasma. We prepared Proteinase K with two wash buffers (WBI) in DNA sample preparation kit. Then, we mixed the plasma with 260 μL Proteinase K and 2.1 mL DNA PBB (binding buffer), and incubated at room temperature for 25 minutes. After that we mixed 500 μL isopropanol with the lysate and then transferred into the High Pure Extender Assembly. Then, these assemblies were centrifuged at 4000 × g for 1 min. The DNA was eluted in 100 μL DNA EB (elution buffer). The extraction yields high quality DNA suitable for further analyses.

RETRACTED

It is noteworthy in the first and second step the data collections were repeated after one day for each subject in order to examine the reproducibility of the results from experiments.

The anti-cancer drug which was used in this research was Cisplatin. Cisplatin as an alkylating agent is widely used for treatment of many cancers such as small and non-small cell lung, prostate, breast, cervical, stomach cancers. The drug was given to patients through a cannula which put into a vein in patient’s arm under the supervision of medical doctor in order to control the experiments and prevent the drug side effects. As we choose the patients from the similar ages, height and weight as well as general health condition, the same dose (80 *mg*/*m*^2^) of Cisplatin was given to all patients.

### Data Analysis

In order to do the analysis, in the first step using the written codes in MATLAB, the values the Hurst exponent and fractal dimension for damaged DNA walk are computed and spectrum of each measure is generated in case of each subject. Then, in order to predict the DNA walk behaviour after using anti-drug cancer, a set of codes was written in MATLAB. Using the properties of damaged DNA walk as input to Equation (13) these codes compute the DNA walk as output. Then, the program computes the Fractal dimension and Hurst exponent in case of each subject. The program also compute the Hurst exponent and Fractal dimension of DNA walk for normal cells in case of each subject.

The value of *F*_0_ is taken as the value of the last point in the spectrum of damaged DNA walk. The initial value of *H* in Equation (13) is the last value of the Hurst exponent in the Hurst exponent plot of damaged DNA.

It is noteworthy that computation of the Hurst exponent in each step was based on Rescaled Range Analysis method which is widely used by statisticians.

Also, as it was mentioned before the anti-cancer drug is modelled as a single Gaussian pulse in this research. So by inserting all required parameters, the DNA walk and it’s related Fractal dimension and Hurst exponent plots are generated in nucleotide distances. The required parameters are brought in Table 1. It is noteworthy that the values of parameters in Gaussian pulse can be changed based on the type, strength and dose of different anti-cancer drugs application.

RETRACTED

## Result

The means of the Hurst exponent variations for the real versus modelled DNA walks in case of 50 subjects are shown in Fig. 5. It is clear that in all cases the modelled DNA walk has smaller values of the Hurst exponent than the real normal DNA walk. As it can be seen in all cases there are small differences between the Hurst exponents for the modelled and real DNA walks. The maximum difference is in case of subject 45 which is 0.05 and indicates for 4.93% difference on average between the real and modelled DNA walk. The average of differences between the Hurst exponent of real and modelled DNA walks is 0.023 which indicates for 3.21% difference on average between the real and modelled DNA walks.

For the better comparison the means of the Fractal dimension variations for the real versus modelled DNA walks in case of 50 subjects are shown in Fig. 6. It is clear that in all cases the modelled DNA walk has bigger values of the Fractal dimension than the real normal DNA walk. As it can be seen in all cases there are small differences between the Fractal dimension for modelled and real DNA walks. The maximum difference is in case of subject 45 which is 0.05.

The analyses of the Hurst exponent and Fractal dimension plots for the modelled and real DNA walks showed that the Fractional Diffusion Model could predict the DNA walk after the application of anti-cancer drug with very high accuracy. In fact, comparing the Hurst exponent and Fractal dimension spectra in case of modelled versus real DNA walk (for healthy cells) give us a very useful tool for examining the strength of the proposed model. Almost in all cases the characteristics of modelled DNA walk are similar with the real DNA walk.

## Discussion

In this research we proposed a new method for forecasting of DNA walk after the application of anti-cancer drug. In this method we built a new model based on Fractional Diffusion Equation (FDE) which makes a relationship between diffusion of drug in tumor and DNA walk as fractal series. In order to test this model the damaged DNA walks for fifty subjects with lung cancer were given to the model and then this model predicted the DNA walks. In order to test the strength of prediction we compared the modelled DNA walk and the real normal DNA walk by computing the Hurst exponent and Fractal dimension spectra of these walks. The analyses showed that Hurst exponent and Fractal dimension spectra for the modelled DNA walks closely resemble the Hurst exponent and Fractal dimension spectra for the real DNA walk respectively. The mean of differences between the modelled and real values was 0.023 which indicates for 3.21% difference on average between the real and modelled DNA walks. This result stands for very high accuracy of the modelling method.

RETRACTED

Here we test the efficiency of our method in case of the special drug and cancer. In fact, the dose of drug application can be changed and the effect of this change in the real experiment compared with the results from mathematical model. Also, the developed model can be applied in case of different drugs (with varying dosage) which are used for treatment of different types of cancer. On the other hand, the simultaneous application of drugs to patients can be studied using this model. So, the proper drug(s) with the required dosage can be advised based on the modelling outcome and considering the patient’s general health condition. Another outcome of this model is its predictability which helps physicians in order to anticipate the future of cancer treatment after drugs application. So, this method can speed up clinical practice for cancer patients and drug, design development and therapy for cancer drugs.

## Additional Information

**How to cite this article**: Namazi, H. *et al.* Mathematical Modelling and Prediction of the Effect of Chemotherapy on Cancer Cells. *Sci. Rep.* **5**, 13583; doi: 10.1038/srep13583 (2015).

## Figures and Tables

**Figure 1:** Drug delivery, diffusion and consumption in tumor.

**Figure 2:** The real damaged DNA walk and solution of Equation (13) (after *l* = 4.2).

**Figure 3:** Hurst exponent plot for the real damaged DNA walk and solution of Equation (13) (after *l* = 4.2).

**Figure 4:** Fractal spectrum plot for the real damaged DNA walk and solution of Equation (13) (after *l* = 4.2).

**Figure 5:** Means of Hurst exponent variation for real and modelled DNA walks in case of different subjects.

**Figure 6:** Means of Fractal dimension variation for real and modelled DNA walks in case of different subjects.

**Table 1:** Values of required parameters.

Variable	Value
*D*	22.41 ± 5.63 *μm*^2^/*s*
*C*	0.3 *m*/*s*
*φ*_0_(*η*,*l*)	1.2
l*	0.003
*σ*	0.0015
